# Perioperative Nursing Management of Patients Undergoing Laparoscopic Ovarian Cystectomy Guided by Ultrasound Imaging under Intelligent Algorithm

**DOI:** 10.1155/2022/7193005

**Published:** 2022-05-04

**Authors:** Shuanghong Lin, Yi Zhao, Dan Lei, Qiongfang Mei, Honggui Fang, Li Wang

**Affiliations:** ^1^Department of Nursing, Hubei No. 3 People's Hospital of Jianghan University, Wuhan, 430033 Hubei, China; ^2^Department of Obstetrics and Gynecology, Hubei No. 3 People's Hospital of Jianghan University, Wuhan, 430033 Hubei, China

## Abstract

This study was aimed at exploring the application value of ultrasonic imaging-guided laparoscopic ovarian cystectomy after denoising by intelligent algorithms in perioperative nursing intervention of patients. In this study, convolutional downsampling was introduced to the UNet model, based on which the residual structure and Recon module were added to improve the UNet denoising model, which was applied to 100 patients who underwent ultrasound imaging-guided laparoscopic ovarian cystectomy. The patients were grouped into a control group receiving conventional nursing and an experimental group receiving perioperative nursing management. The various experimental indicators were comprehensively evaluated. The results revealed that after denoising using the improved UNet model, the ultrasound image showed no unnecessary interference noise, and the image clarity was significantly improved. In the experimental group, the operation time was 55.45 ± 6.13 days, the intraoperative blood loss was 71.52 ± 9.87 days, the postoperative exhaust time was 1.9 ± 0.73 days, the time to get out of bed was 1.2 ± 0.85 days, the complication rate was 8%, the hospitalization time was 7.3 ± 2.6 days, and the nursing satisfaction rate reached 98%. All above aspects were significantly better than those of the control group, and the differences were statistically significant (*P* < 0.05). In short, the improved UNet denoising model can effectively eliminate the interference noise in ultrasound and restore high-quality ultrasound images. Perioperative nursing intervention can accelerate the recovery speed of patients, reduce the complication rate, and shorten the length of stay in hospital. Therefore, it was worthy of being widely used in clinical nursing.

## 1. Introduction

Ovarian cyst is a kind of ovarian tumor in a broad sense. Although it affects women of all ages, it is more common for women aged 20-50 [1]. Ovarian tumors are common tumors in female reproductive organs. They have a variety of characteristics and morphologies, such as single or mixed, unilateral or bilateral, vesicular or substantial, and physiological or pathological [2, 3]. Physiological ovarian cysts will disappear on their own due to the periodic changes of the ovaries. However, in some cases, the follicles and corpus luteum cysts grow too fast and the ovarian tissue splits, causing bleeding. Because there is no outlet, the blood is wrapped in the ovaries, forming a hematoma [4]. However, whether it is a cyst or a hematoma, it will gradually shrink and disappear naturally within a few months. If there is a situation that does not shrink but increases (above 6 cm in diameter), or if it is a cyst in a prepubertal girl or post-menopausal woman, the possibility of ovarian tumors must be suspected and diagnosis and treatment are required [5, 6].

Traditional ovarian cyst excision and laparotomy bring greater pain and injury to patients, slower incision healing, longer hospital stay, and higher risk of complications [7, 8]. At present, laparoscopic minimally invasive surgery guided by ultrasound is commonly used in clinical practice, which causes little trauma to the patient and fast recovery after surgery. It is increasingly used in the field of gynecological surgery and is considered to be “Golden operation” to remove benign ovarian cysts [9]. However, in the process of ultrasound imaging, a large number of scattered waves will be generated due to the propagation of ultrasonic waves. When they meet in space, they will cause constructive and destructive interference, resulting in bright and dark spots, that is, speckle noise. These noises will reduce the quality of ultrasound imaging and will have a great impact on clinical applications [10, 11]. This requires the use of intelligent algorithms for denoising.

The traditional image denoising algorithm requires artificial prior information, its generalization is not strong, and the denoising effect is not good [12]. In recent years, the application of deep learning in the medical field has become more and more extensive. It is an important subject in the field of artificial intelligence and a new research direction in the field of machine learning. It is mainly used in classification or prediction. It can automatically learn the deep-level feature representation of data, which is more accurate than traditional methods [13, 14]. The image denoising algorithm based on deep learning has a flexible structure and strong self-learning ability, which can be used to make up for the shortcomings of traditional image denoising algorithms [15]. In addition, it can not only keep the many details of the ultrasound image intact, but also better remove the noise on this basis, and restore the original high-quality ultrasound image [16], which is beneficial to be used as a guide during surgery.

The whole period from the patient's decision to undergo laparoscopic ovarian cystectomy until the patient is cured, and discharged after the operation is called the perioperative period. Laparoscopic ovarian cystectomy is an invasive treatment process. During the perioperative period, patients will be affected by diseases, anesthesia, and surgery. There are some risks, and it also brings great psychological pressure to patients and their families. Routine nursing measures can improve the patient's nursing effect to some extent, but the effect is still poor. Perioperative nursing intervention is a new nursing model, which is a new standard and new requirement put forward by the clinic in order to enable patients to have a better nursing experience and effect. Therefore, perioperative nursing management is of great significance, which is related to the therapeutic effect of surgery and the recovery of patients after surgery [17].

In this work, a denoising model was constructed based on a deep learning algorithm, which was applied to the ultrasound guidance of laparoscopic ovarian cystectomy in 100 patients. In addition, different nursing intervention methods were given to the two groups of patients. This study was aimed at exploring the application value of ovarian cystectomy and perioperative nursing measures under the guidance of improved UNet algorithm, aiming to provide reliable guidance for the surgical process and postoperative recovery of patients undergoing ovarian cystectomy.

## 2. Materials and Methods

### 2.1. Research Objects

One hundred patients who would be treated in hospital from March 2019 to March 2021 and diagnosed as ovarian cysts by imaging examination were selected, and they underwent ultrasound-guided laparoscopic ovarian cystectomy. The age range was 25-38 years old, with an average age of 29.78 ± 4.36 years old. All patients were randomly divided into a control group and an experimental group, with 50 cases in each group. The patients in the control group were managed by routine nursing, and the patients in the experimental group were managed by nursing during the perioperative period. This study had been approved by the ethics committee of hospital. All experimental-related matters had been informed to the patients, and the informed consent form had been signed.

Inclusion criteria: (1) all types except ovarian malignancies can be included, such as simple cyst, follicular cyst, mesangial cyst, and endometriotic cyst; (2) the diameter of the cysts was less than 15 cm, and all were unilateral; (3) gynecological examination cyst was isolated, cyst pedicle was long, and mobility was good with no adhesion; (4) there were no obvious surgical contraindications (such as excessive cyst and too short ovarian proper ligament); (5) postoperative pathological diagnosis was benign; and (6) menstruation was normal in the periodicity.

Exclusion criteria: (1) patients with a history of ovarian surgery; (2) patients with severe organic diseases; (3) patients with breast, thyroid, adrenal glands, and other diseases; (4) patients with malignant or suspected malignant tumors; and (5) incomplete clinical data or poor compliance.

### 2.2. Denoising Algorithm Based on Improved UNet

In ultrasound imaging, because it is different from general grayscale and color images, the semantics are not complicated and the structure is single, so the semantic features regardless of the level are very critical. In ultrasound imaging, because there are not many data sets, it is not easy to obtain, and it is often necessary to use a targeted network structure when extracting features. The maximum pooling downsampling commonly used in network models constructed based on traditional UNet algorithms will cause excessive loss of image information, and it is not clear when processing edges. Therefore, a network denoising model based on the improved UNet algorithm was proposed in this study.

UNet is an image segmentation network widely used in medical image processing. The process is to input a picture, and the output is the segmentation result of the target. According to the difference between the result and the real segmentation, the segmentation network is back-propagated to train the segmentation network. Its network structure was shown in Figure 1.

As shown in Figure 1 that the left area was used for downsampling feature extraction, and the right area was interpolated upsampling. Jumping connections were used on the same layer to ensure that as many underlying features as possible can be combined in the final imaging to have richer imaging information. UNet structure is sometimes called codec structure. Encoding meant the process of extracting features, while decoding was the process of restoring abstract features back to the template. Introducing jump connections into it can restore high-level semantic features and combine more low-level information at the same time, thereby improving the denoising performance of the network model.

In this study, the concept of residual learning was introduced into the improved network model based on UNet, and the equation for removing noise in ultrasound imaging was shown as follows:

(1) $$\begin{array}{c} a+e=b. \end{array}$$

It was supposed that the noise-containing ultrasound image was *a*, *b* represented the final high-quality noise-free image obtained, and *e* represented the noise distribution in the noise-containing ultrasound image. The noise was learned through the network model of nonresidual structure, and a mapping can be obtained, expressed as the following:

(2) $$\begin{array}{c} R\left(a\right)=b. \end{array}$$

A noise-containing ultrasound image was imported into this function, and the final result was a high-quality image without noise. The noise distribution in this kind of imaging was *D*(*a*) ≈ *e*. When the overall residual learning noise *a* + *e* was close to *b*, it was necessary to update the weight parameters, then the gradient descent method was used here. Minimizing the learning and fitting can maintain a stable state of the entire network. The improved UNet model was based on the UNet structure, added with residual connections, and started to use the residual block structure. The residual block structure was shown in Figure 2.

In the figure above, ⨂ represented the addition of the corresponding elements. The residual block contained two 3 × 3 convolutional layers, PReLU was inserted between them, and the input and output connections were skip connections. The PReLU activation function was expressed as the following:

(3) ReLUa=max0,a.

When *a* was less than 0, the gradient was 0, and the corresponding parameter would stop updating. To make up for this shortcoming, PReLU was introduced, and the following Equation (4) was its general expression equation:

(4) PReLUaf=af,fraf>0,tfaffraf≤0.

In the above equation, *f* represented different channels, and when the gradient was *t*_*f*_ = 0, it would degenerate to ReLU. Although the parameters introduced by PReLU would slightly increase the amount of calculation, the impact was not large, especially when the same gradient was used for different channels, the trouble caused by the parameter amount was negligible.

In the original UNet convolution process, each time the next layer was downsampled, the width and height of the corresponding feature map would be reduced by half, and the number of channels would be doubled. Therefore, the RDUB module was introduced in this study, which can convert the feature map under the initial structure into the residual block structure, and copy and splice it to supplement the underlying information by superimposing the feature map.

In order to restore as much image feature information as possible, the Recon module was introduced after the RDUB module, and these conditions were combined to build an improved UNet denoising model to deal with the noise contained in ultrasound imaging. The basic structure of the improved UNet denoising model was shown in Figure 3.

In the improved UNet model, jump connections were still used to connect the bottom layer and deep layer feature maps, so that the bottom layer feature information can be retained as much as possible, and the output high-quality ultrasound image can be obtained.

The quantitative evaluation indicators of ultrasound images included peak signal to noise ratio (PSNR) and structural similarity (SSIM). The performance of the model was measured by the PSNR value, in dB.

(5) $$\begin{array}{c} \text{PSNR}=10\log_{10}\left(\frac{{\left(2^{n}-1\right)}^{2}}{\text{MSE}}\right). \end{array}$$

In the above equation, MSE represented the mean square error between the original image *X* and the reference image *Y*. The larger the PSNR value, the smaller the distortion.

SSIM is a measure of the similarity of two images, which can be used to evaluate the quality of the processed images, expressed as follows:

(6) $$\begin{array}{c} \text{SSIM}\left(X,Y\right)=\frac{\left(2u_{X}u_{Y}+C_{1}\right)\left(2\sigma_{XY}+C_{2}\right)}{\left({u_{X}}^{2}+{u_{Y}}^{2}+C_{1}\right)\left({\sigma_{X}}^{2}+{\sigma_{Y}}^{2}+C_{2}\right)}. \end{array}$$

In Equation (6) above, *u*_*X*_ and *u*_*Y*_ referred to the mean values of *X* and *Y*, respectively; *σ*_*X*_ and *σ*_*Y*_ represented the standard deviations; and *C*_1_ and *C*_2_ were constants.

### 2.3. Nursing Method

For patients in control group, the conventional nursing method was adopted. Specifically, it included the use of psychological nursing for patients to calm their nervousness. It should provide a quiet and comfortable ward environment suitable for postoperative recovery, pay attention to indoor ventilation, closely observe the changes in the patient's body temperature, coagulation function and other indicators after surgery, and change the incision dressing frequently to reduce the chance of complications. In addition, it had to pay attention to diet nursing, fasting milk, beans, and other high-protein foods before surgery. A liquid diet was the best, and proper nutrition should be enhanced after surgery to help recovery.

For patients in experimental group: the perioperative nursing management method was adopted. I. Preoperative nursing included below aspects. The patient's emotional and mental state was evaluated comprehensively. A personalized nursing plan was developed according to the evaluation results. Professional nurses communicated with patients patiently, fully understood the patient's mood before undergoing the operation, and answer related questions raised by the patient. At the same time, the popularization of surgical knowledge was introduced, so that patients can learn about laparoscopic ovarian cystectomy, the successful cases, and success rate of the operation, and relieve the nervousness of the patients. The patient was informed about the preoperation precautions such as fasting within 12 hours before the surgery and makes adequate preparations before the surgery. II. Postoperative nursing was introduced as follows. After the surgery, the patient was returned to the ward, and the rehabilitation environment should be quiet and comfortable. It should closely observe the patient's vital signs and report to the doctor if there is any abnormality. Professional nursing staff would perform posture nursing for the patient. After the patient recovered from anesthesia, the patient was helped to inhale oxygen and do appropriate rehabilitation training to reduce the chance of complications and minimize the length of stay in hospital. It was also necessary to plan a reasonable diet plan for the patient. After the surgery, the patient should eat more high-protein, high-fiber foods, and fresh fruits and vegetables to help the body recover.

### 2.4. Ultrasound-Guided Laparoscopic Ovarian Cystectomy

The patient was fully prepared before the surgery, confirmed that there was no contraindication to the operation, expressed the knowledge of the operation risk, and signed the informed consent form. The patient emptied the urine stored in the bladder and lay flat on the examination bed of the ultrasound intervention operation room. The patient took the position of the lithotomy, and determined the location of the cyst and measured the size of the cyst through ultrasound, which was based on the improved UNet algorithm for denoising, to confirm the presence of blood flow signals in and around the cyst. The patient underwent general anesthesia with tracheal intubation, and laparoscopic system was used. It should routinely disinfect the drape to ensure that the umbilicus was clean. A longitudinal incision about 8-10 mm above the umbilicus was made, the pneumoperitoneum needle was punctured into the abdominal cavity, and a 10 mm pipe-like working channel was taken from the incision and pierce it above the umbilicus to insert the mirror body. A 10 mm incision was made at the position of about two transverse fingers on the upper edge of the anterior superior iliac spine of the patient's left lower abdomen, a 10 mm duct-like working channel was inserted, a 5 mm incision was made at the McGill point of the right lower abdomen, and a 5 mm working channel was inserted.

It should carefully explore the pelvic cavity and abdominal cavity to confirm whether there were abnormalities such as cysts and adhesions, separate the adhesion tissue, and restore the basic anatomical structure of the organs. The laparoscopic puncture needle was injected into the middle part of the cyst and the ovarian cortex at the position away from the pelvic ligament of the ovary and the ovarian hilum, and the syringe was connected to push in the diluted pituitary gland. The tissue forceps was adopted to fix the ovary, and the ovarian cortex was cut to find the gap between the ovarian cyst wall and normal ovarian tissue, and distinguish the level. The cyst tissue was separated with a tearing method. The wall of the cyst was mostly grayish-yellow, while the normal ovarian tissue was pink. The cyst was removed from the clear margins, and it should ensure that the cyst was completely removed while trying not to lose too much of the normal cortical tissue.

After the cyst fluid flowing out of the cyst rupture was sucked up, it was repeatedly washed with normal saline. The low-power bipolar electrocoagulation was used to stop bleeding, and the ovarian tissue was continuously sutured with absorbable sutures. The cyst tissue was taken out, and the pelvic cavity was washed repeatedly with normal saline. After it was confirmed that there were no abnormalities such as blood oozing, an abdominal drainage tube was placed, the abdominal cavity was exhausted, and the abdomen was extubated and closed. Anti-inflammatory and hemostatic drugs were routinely given after surgery.

### 2.5. Evaluation Criteria

The operation time, intraoperative blood loss, postoperative exhaust time, time to get out of bed, the occurrence of complications, the incidence rate, and patients' satisfaction with nursing were observed and recorded in the control group and the experimental group. Nursing satisfaction was calculated using a self-made questionnaire. Very satisfied: more than 80 points; satisfied: 60-80 points; dissatisfied: less than 60 points. Total satisfaction (%) was calculated with below equation: (number of people with very satisfied result + number of people with satisfied result)/number of respondents.

### 2.6. Statistical Analysis

All data were statistically analyzed using SPSS 24.0 software, and measurement data were expressed as mean standard deviation ($\overset{¯}{x}\pm s$). The data comparison before and after the surgery within the group used the *t* test, and the comparison between the two groups used the two-sample *t* test. *P* < 0.05 meant the difference was statistically significant.

## 3. Results

### 3.1. Ultrasound Imaging Noise Reduction Experiment

Denoising experiments were performed on ultrasound images using four different methods. As shown in Tables 1 and 2, the average PSNR and SSIM results of the improved UNet algorithm selected in this work were better than those of other algorithms, and the denoising effect was better.

### 3.2. Comparison on Ultrasound Images before and after Using the Improved UNet Algorithm

Figure 4 below was an ultrasound image of a patient in the experimental group who was admitted to the hospital with a complaint of “left ovarian serous cystadenoma” 3 months ago. From the ultrasound image, it can be observed that there was a cystic dark area in the appendage area on the left side of the patient, with small light spots floating, and ovarian tissue echoes. However, the ultrasound image contained extra speckle noise, and the image quality was low. After the improved UNet algorithm was adopted for denoising, the quality of ultrasound images was significantly improved, and there was no interfering noise, which was conducive to the judgment of the condition.

### 3.3. Comparison of General Clinical Data between the Two Groups of Patients

As shown in Table 3, there was no significant difference between the control group and the experimental group in terms of average age, height, weight, cyst diameter, course of disease, and pathological classification of cysts, which were not statistically significant (*P* > 0.05), showing comparability.

### 3.4. Comparison of the Treatment of the Two Groups of Patients

On the operation time, the average time taken by the patients in the experimental group was 55.45 ± 16.13 minutes, which was shorter than that (60.83 ± 17.62 minutes) in the control group. In terms of intraoperative blood loss, patients in the experimental group were 71.52 ± 9.87 mL, which was less than that (78.54 ± 10.02 mL) in the control group. The postoperative exhaust time of patients in the experimental group was 1.9 ± 0.73 days, which was shorter than that (2.3 ± 0.84 days) in the control group. Patients in the experimental group can get out of bed after 1.2 ± 0.85 days, while patients in the control group needed 1.7 ± 0.91 days. There were significant differences between the two groups (*P* < 0.05). The details were shown in Figures 5, 6, and 7.

### 3.5. Comparison of Complication Rate between Two Groups of Patients

Among the postoperative complications (bleeding, subcutaneous emphysema, pain, nausea and vomiting, infection, high fever, abdominal distension, and back soreness), the numbers of patients in the control group were 2 cases, 0 cases, 1 case, 1 case, 1 case, 2 cases, 1 case, and 0 case; while those in the experimental group were 1 case, 0 case, 1 case, 0 case, 0 case, 1 case, 0 case, and 1 case. The probability of complications in the experimental group was 8%, which was significantly lower than the 16% in the control group. The difference was statistically significant (*P* < 0.05). It can check the Figures 8 and 9 below for details.

### 3.6. Comparison of the Length of Stay in Hospital between the Two Groups

As shown in Figure 10, the average length of stay in hospital of patients in the experimental group was 7.3 ± 2.6 days, which was significantly less than the 9.5 ± 2.8 days of patients in the control group. The difference was statistically significant (*P* < 0.05).

### 3.7. Comparison of Nursing Satisfaction between the Two Groups of Patients

In nursing satisfaction, 69% of patients in the control group were very satisfied, 24% were satisfied, and 7% were dissatisfied. In the experimental group, 76% of patients were very satisfied, 22% were satisfied, and 2% were dissatisfied. The total satisfaction degree of the experimental group was 98%, which was significantly higher than the 93% of the control group, and the difference was statistically significant (*P* < 0.05). It could check Figure 11 for details.

## 4. Discussion

For malignant tumors such as ovarian cysts, which can seriously endanger women's health, they have reached the middle or advanced stage when they are found, so timely treatment is required [18]. Ultrasound-guided laparoscopic ovarian cystectomy used in this work was a minimally invasive surgical method that is widely used. It can accurately locate and remove ovarian cysts, which meets the requirements of patients, especially young women, for more minimally invasive surgery, with less surgical trauma and faster postoperative recovery [19]. However, ultrasound imaging inevitably has some shortcomings such as noise interference and low image quality. This is because ultrasound is imaged using ultrasound signals reflected by biological tissue. Under the influence of constructive and destructive interference, the final ultrasound will have Gaussian noise or speckle noise and other interference factors [20, 21], which affects the reading and the doctor's judgment on the patient's condition.

The traditional algorithm will cause too much loss of image information during denoising, and the effect is not good, and it cannot automatically adjust parameters, resulting in low work efficiency. In recent years, deep learning has rapidly developed into a research hotspot in medical image analysis, which can automatically localize implicit disease diagnosis features from medical image big data [22]. In this work, convolutional downsampling was introduced into the UNet network model to replace the original max pooling downsampling, and a residual structure and a Recon module were added to it. The improved UNet network denoising model based on the above conditions was used to improve the noise problem of ultrasound imaging. At the same time, nursing management before and after surgery also plays an important role in the perioperative period of patients. In this work, 100 patients who underwent ultrasound-guided laparoscopic ovarian cystectomy were selected and randomly divided into a control group of 50 cases of conventional nursing and an experimental group of 50 cases of perioperative nursing management. In the experimental group, on the basis of conventional nursing, professional nursing staff performed nursing interventions on patients before and during the surgery, as well as nursing in psychological and dietary aspects. The results showed that the image denoising PSNR and SSIM values of the improved UNet algorithm were better than NL-mean, CNN, and UNet algorithms; there was no extra interference noise in the denoised ultrasound image; and the image clarity was significantly improved. Such results were consistent to Mei et al. [23]. It indicates that the improved UNet denoising model can effectively remove speckle noise in images and restore high-quality ultrasound images. The innovation of this work was to use ultrasound based on the improved UNet algorithm as a surgical guide for ovarian cystectomy, so as to explore its clinical value. The experimental group was better than the control group in terms of treatment (operation time, intraoperative blood loss, postoperative exhaust time, and time to get out of bed), complication rate, hospital stay, and nursing satisfaction (*P* < 0.05). It suggests that under the perioperative nursing management, the patient's surgical condition and postoperative recovery effect are more ideal, which was also mentioned in the article by He et al. in 2021 [24]. Perioperative nursing intervention for patients undergoing ovarian cystectomy can improve the recovery speed of patients, reduce the incidence of complications, and shorten hospitalization time, so it could be promoted and applied.

## 5. Conclusion

In this study, 100 patients who met the requirements were selected and divided into a conventional nursing control group and a perioperative nursing intervention experimental group. At the same time, an improved UNet denoising model was constructed based on the UNet structure and applied to ultrasound-guided laparoscopic ovarian cystectomy. The results proved that the ultrasound image was denoised by the improved UNet model without unnecessary interference and noise, and the image clarity was improved. The experimental group was significantly better than the control group in terms of operation time, intraoperative blood loss, postoperative exhaust time, the time to get out of bed, complication rate, length of stay in hospital, and nursing satisfaction, showing statistically significant differences (*P* < 0.05). The disadvantage was that due to the limited conditions, the number of patients in this study was small, and the experimental results had some limitations and one-sidedness. In the future, the sample size would be expanded, and more in-depth research would be conducted in this direction to provide a reference for the clinical treatment and nursing of patients with ovarian cysts.

## Figures and Tables

**Figure 1:** Structure of UNet.

**Figure 2:** Structure of residual block.

**Figure 3:** The basic structure of improved UNet denoising model.

**Figure 4:** Comparison of ultrasound imaging results before and after optimization of the improved UNet algorithm. (a) was the original ultrasound image; (b) was the ultrasound image denoised by the improved UNet algorithm.

**Figure 5:** Comparison of operation time between the two groups of patients. ∗ indicated that the operation time of the experimental group was statistically significant compared with that of the control group (*P* < 0.05).

**Figure 6:** Comparison of intraoperative blood loss between the two groups of patients. ∗ indicated that the intraoperative blood loss of the experimental group was statistically significant compared to the control group (*P* < 0.05).

**Figure 7:** Comparison of postoperative exhaust time and the time to get out of bed between the two groups of patients. ∗ indicated that the postoperative exhaust time and the time to get out of bed in the experimental group were statistically significant compared to the control group (*P* < 0.05).

**Figure 8:** Comparison of the number of complications between the two groups. (a) represented the comparison on numbers of patients with bleeding, subcutaneous emphysema, pain, nausea, and vomiting; (b) showed the comparison on numbers of patients with infection, high fever, abdominal distension, and back soreness.

**Figure 9:** Comparison of the complication rate of the two groups of patients.

**Figure 10:** Comparison of length of stay in hospital between two groups of patients. ∗ indicated that the length of stay in hospital of the experimental group was statistically significant compared to the control group (*P* < 0.05).

**Figure 11:** Comparison of nursing satisfaction between the two groups of patients. ∗ indicated that the total nursing satisfaction of the experimental group was statistically significant compared with that of the control group (*P* < 0.05).

**Table 1:** PSNR results of different denoising algorithms.

Algorithm	Standard deviation at 0.5	Standard deviation at 1	Standard deviation at 1.5	Standard deviation at 2	Standard deviation at 2.5
NL-mean	33.0834	31.5236	28.9535	28.6321	27.5489
CNN	36.2467	32.7854	30.8535	30.1524	29.4623
UNet	38.2468	34.2478	32.3563	31.3746	30.8624
Improved UNet	38.7367	35.2856	33.2478	32.6909	31.3689

**Table 2:** SSIM results of different denoising algorithms.

Algorithm	Standard deviation at 0.5	Standard deviation at 1	Standard deviation at 1.5	Standard deviation at 2	Standard deviation at 2.5
NL-mean	0.8734	0.7626	0.7368	0.7245	0.6902
CNN	0.9768	0.9345	0.9103	0.8835	0.8523
UNet	0.9624	0.9533	0.9247	0.9024	0.8965
Improved UNet	0.9876	0.9631	0.9428	0.9257	0.9025

**Table 3:** Comparison of general clinical data of the two groups of patients.

Essential information	Control group	Experimental group	Statistic value	*P* value
Average age (years old)	29.56 ± 3.78	29.37 ± 4.12	1.578	0.674
Weight (kg)	63.82 ± 8.03	62.57 ± 7.45	1.428	0.586
Height (cm)	162.88 ± 5.06	161.33 ± 5.41	0.953	0.742
Cyst diameter (mm)	68.731 ± 6.76	69.34 ± 7.28	0.648	0.721
Course of disease (months)	9.2 ± 1.5	9.3 ± 1.7	1.753	0.633
Serous cyst (people)	9	8	1.698	0.725
Mucinous cyst (people)	7	8	2.854	0.544
Chocolate cyst (people)	10	11	1.649	0.631
Simple cyst (people)	4	3	1.535	0.578

## Data Availability

The data used to support the findings of this study are available from the corresponding author upon request.

## References

[1] Henes M., Engler T., Taran F. A. (2018). Ovarian cyst removal influences ovarian reserve dependent on histology, size and type of operation. *Women’s Health*.

[2] Nowak-Psiorz I., Ciećwież S. M., Brodowska A., Starczewski A. (2019). Treatment of ovarian endometrial cysts in the context of recurrence and fertility. *Advances in Clinical and Experimental Medicine*.

[3] Choy K. T., Kumar K., Ratnapala D. (2020). Retroperitoneal schwannoma masquerading as an ovarian cyst. *ANZ Journal of Surgery*.

[4] Pal S., Kumari P., Jain A., Sinha S. K. (2020). Fetal ovarian cyst managed laparoscopically in the neonatal period. *Indian Pediatrics*.

[5] Llorens Salvador R., Sangüesa Nebot C., Pacheco Usmayo A., Picó Aliaga S., Garcés Iñigo E. (2017). Neonatal ovarian cysts: ultrasound assessment and differential diagnosis. *Radiologia*.

[6] Xiang H., Han J., Ridley W. E., Ridley L. J. (2018). Fishnet/cobweb ovary: haemorrhagic ovarian cyst. *Journal of Medical Imaging and Radiation Oncology*.

[7] Nii M., Kondo E., Maki S. (2018). Safety and efficacy of laparoscopic oophorocystectomy for ovarian dermoid cyst associated with autoimmune hemolytic anemia. *Gynecology and Minimally Invasive Therapy*.

[8] Liu X., Song J., Zhang Y., Zhang Y., Hu X. (2021). Different doses of nalbuphine combined with dexmedetomidine in laparoscopic oophorocystectomy. *Medical Science Monitor*.

[9] Hernandez-Nieto C., Lee J. A., Gonzalez K., Mukherjee T., Copperman A. B., Sandler B. (2020). Conservative treatment versus surgical excision of ovarian dermoid cysts: impact on ovarian stimulation and IVF cycle success. *International Journal of Gynaecology and Obstetrics*.

[10] Radosz J., Pleban D. (2018). Ultrasonic noise measurements in the work environment. *The Journal of the Acoustical Society of America*.

[11] Bevan R. L. T., Zhang J., Budyn N., Croxford A. J., Wilcox P. D. (2019). Experimental quantification of noise in linear ultrasonic imaging. *IEEE Transactions on Ultrasonics, Ferroelectrics, and Frequency Control*.

[12] Gao F., Li B., Chen L., Wei X., Shang Z., He C. (2020). Ultrasonic signal denoising based on autoencoder. *The Review of Scientific Instruments*.

[13] Yan Z., Xu X., Wang Y. (2021). Application of ultrasonic Doppler technology based on wavelet threshold denoising algorithm in fetal heart rate and central nervous system malformation detection. *World Neurosurgery*.

[14] Dai M., Li S., Wang Y., Zhang Q., Yu J. (2019). Post-processing radio-frequency signal based on deep learning method for ultrasonic microbubble imaging. *Biomedical Engineering Online*.

[15] Cai Y., Song Y., Ni P., Liu X., Li X. (2021). Subwavelength ultrasonic imaging using a deep convolutional neural network trained on structural noise. *Ultrasonics*.

[16] Engelman D. T., Ben Ali W., Williams J. B. (2019). Guidelines for perioperative care in cardiac surgery. *JAMA Surgery*.

[17] Al-Niaimi A., Alyami M., Balonov K. (2020). Guidelines for perioperative care in cytoreductive surgery (CRS) with or without hyperthermic intraperitoneal chemotherapy (HIPEC): enhanced recovery after surgery (ERAS®) society recommendations -- part I: preoperative and intraoperative management. *European Journal of Surgical Oncology*.

[18] Bachmann F., Glander P., Budde K., Bachmann C. (2018). High incidence of ovarian cysts in women receiving mTOR inhibitors after renal transplantation. *Journal of Women's Health (2002)*.

[19] Boos J., Brook O. R., Fang J., Brook A., Levine D. (2018). Ovarian cancer: prevalence in incidental simple adnexal cysts initially identified in CT examinations of the abdomen and pelvis. *Radiology*.

[20] Wang Z., Cheng J. (2021). Numerical and analytical study for ultrasonic testing of internal delamination defects considering surface roughness. *Ultrasonics*.

[21] Li D., Fei C., Zhang Q., Li Y., Yang Y., Zhou Q. (2018). Ultrahigh frequency ultrasonic transducers design with low noise amplifier integrated circuit. *Micromachines*.

[22] Kovács G., Nagy S. (2020). Ultrasonic sensor fusion inverse algorithm for visually impaired aiding applications. *Sensors*.

[23] Mei Y., Jin H., Yu B., Wu E., Yang K. (2021). Visual geometry group-UNet: deep learning ultrasonic image reconstruction for curved parts. *The Journal of the Acoustical Society of America*.

[24] He M., Tong L., Zou Y., Li Z. (2021). Effect of 5A nursing mode combined with fine nursing management on perioperative self-efficacy and living quality of hysteromyoma. *American Journal of Translational Research*.

